The article "Stimulating Brand Innovation Strategy via Knowledge Acquisition, Market Orientation, and Strategic Capability Using Social Media Within China’s Online Technology Industry" was retracted in 2025. Reasons: unreliable results or conclusions; a conflict of interest; concerns about the peer review; concerns about the citations.

# Stimulating Brand Innovation Strategy *via* Knowledge Acquisition, Market Orientation, and Strategic Capability Using Social Media Within China’s Online Technology Industry

**DOI:** 10.3389/fpsyg.2022.860307

**Published:** 2022-03-14

**Authors:** Yaliu Yang, Xiaowei Zheng

**Affiliations:** ^1^Business School, Suzhou University, Suzhou, China; ^2^Department of International Trade, Dong-A University, Busan, South Korea

**Keywords:** social media, brand innovation, strategic capability, knowledge acquisition, market orientation, proactive, responsive, China

## Abstract

In the context of China’s online technology business, this study explores the linkages between knowledge acquisition *via* social media, two modes of market orientation (proactive and responsive), social media strategic capability, and brand innovation strategy. Data were collected from 853 Chinese technology firms with the help of questionnaire. To analyze the collected data structure, equation modeling was applied using smart-PLS 3.3 version. Results indicate that knowledge acquisition from social media, market orientation (proactive and responsive), and strategic capability has significant impact on brand innovation in the context of social media. Furthermore, strategic capability on social media moderates the relationship between knowledge, market orientation (proactive and responsive), and brand innovation in the context of social media. This study offers new perspectives on market orientation and brand innovation strategy by extending the literature and testing key assumptions. Moreover, using social media knowledge in social media marketing and innovation management is a sensible approach for making changes and transforming an organization.

## Introduction

Social media usage is booming as marketers find new ways to reach consumers. Businesses can interact directly with their customers through social media, engage with them, and amplify their voices. Unfortunately, companies are still unsure how to effectively utilize social media. Social media strategies often focus on platforms as separate entities rather than interrelating to form a coherent whole. With its constant changes, social media requires an even more holistic approach (Cai et al., 2015).

Social media marketing has been extensively researched in recent years. Social media initiatives and brand innovations are among the topics explored in this study, including how to acquire knowledge from social media, strategic capabilities when using social media, market orientation, and how to use social media for brand innovation (Muduli and Trivedi, 2020; Gupta and Syed, 2021). Despite this, the research on the topic is rarely accompanied by a strategic perspective. Social media is particularly effective in driving marketing strategies when firms use it. It is rare for a holistic empirical view of social media as a strategic marketing platform in the literature (Pang, 2021).

Research on social media market knowledge and subsequent innovations lacks a comprehensive understanding of how it contributes to market orientation and brand innovation. Two of the essential firm-level activities and drivers of economic development, according to researchers, are the acquisition of knowledge and the direction of the company on the market (Zhao et al., 2019). In examining, how companies are inspired by social media knowledge to become more informed about market opportunities and become more market-oriented, such as in their relationship with clients and competitors, an understanding of the processes of acquiring social media knowledge, and how it is used in organizations can be provided (Wang et al., 2016).

Literature review indicates that most firms are motivated to discover market opportunities by either being proactive or responsive (Duffett, 2015; Gul et al., 2021a). A responsive market orientation organization meets customers’ needs within the existing market structure in response to customer preferences. In contrast, proactive market orientation speaks to latent customer needs, i.e., those that are not explicit and simply not conscious of. These orientations are, however, found to affect innovation differently (Hanusch and Tandoc, 2019; Geissinger et al., 2021). Furthermore, these topics are seldom researched in transitional economies, and they are rarely applied to social media. By examining how market orientation, knowledge acquisition, and brand innovation in China’s dynamic social media environment contribute to new online ventures, we aim to bridge this knowledge gap (Salo, 2017; Gul et al., 2021b).

We examine the direct impact of social media on these relationships since research indicates that the strategic capability plays a direct and moderating role in the above relationships. A unique opportunity presents itself to assess the impact of social media branding in China when the Chinese economy is undergoing structural change (Chen et al., 2020; Jamil et al., 2022). To better understand the effect of social media knowledge acquisition and market orientation on innovative brand strategies, we intend to analyze the influence of social media on new online technology ventures. According to our model, we rely on the theory of social capital, which stresses the benefits of information flow within social networks and reciprocal cooperation among them. Accordingly, the research will examine organizations’ social media strategic capabilities, namely, their ability to integrate social media skills, resources, and knowledge into strategic planning. During this study, we examined the impact of innovation on social media strategic capabilities, which is, according to our understanding, the first of its kind. The knowledge acquired through social media can determine how effective an organization is at managing its brand. Failure by industrial marketers to recognize the importance of social media knowledge will lead to a drop in market and customer awareness, which will erode both innovation and innovation landscapes and a critical source of brand innovation.

## Literature Review and Hypotheses Development

### Using Social Media for Knowledge Acquisition and Brand Innovation

The use of social media facilitates knowledge acquisition, searching for knowledge, discovery, and transfer of knowledge. Getting the most out of every knowledge resource at a firm’s disposal and transforming it into activities that create value is what determines its performance. The importance of knowledge acquisition is highlighted by Geissinger et al. (2021) regarding new technology ventures. Companies with limited resources and dynamic environments must gain knowledge of the external environment through social media to succeed with brand innovation. Khan et al. (2021) argue that knowledge acquisition plays a vital role in a positive performance and the quality of innovation. Kaimkhani (2018) pointed out that acquiring knowledge makes it easier to understand a wide range of information, making it easier to develop innovative products or processes to meet market needs. According to Wang et al. (2016), the development of technology relies on two factors associated with knowledge acquired from external relationships. Knowledge increases the capabilities of the organization. In addition, knowledge can be utilized to develop technologies that differentiate organizations from each other. New technology firms must constantly learn and adapt to new technologies and markets to create new products and improve in response to dynamic social media environments.

Durana et al. (2021) showed that you have a better chance of enjoying the benefits of traditional sales approaches if you adjust your attitude to one that relies on industry and market knowledge. With the support of exploitative or exploratory learning characteristics, organizations can improve their positioning strategy by participating in the dissemination and production of knowledge about their competitors and consumers (Kovacova and Lăzăroiu, 2021; Valaskova et al., 2021). People believe these skills or methods of learning are critical to success in the marketplace. The concept has been discussed extensively in a variety of business and marketing texts. Competitive advantage is most often gained through resource combination and resource switching, with capabilities serving as the primary means by which this is accomplished. Resource advantage theory and market orientation are both relevant here (Matkevičienė and Jakučionienė, 2021).

Often, knowledge is gained by interacting with external stakeholders. Companies can accurately evaluate new opportunities, information, and added value with such knowledge. Having more knowledge makes companies more capable of strategically orienting their products and differentiating them (Chen et al., 2020; Gul et al., 2021c). If multiple resources and processes are available, it is easier to recombine existing information and ideas to develop more innovative solutions. A substantial repository of knowledge related to the task may be required to create innovative solutions and achieve goals. The acquisition of new technologies allows companies to change how they manufacture new products by using new raw materials (Al-Maroof et al., 2021). Knowing the market, customers’ preferences, distribution channels, and production methods are better understood. Companies can develop or improve products based on evolving market demands using their expertise in new and innovative ways using such information (Awan et al., 2021a). Therefore, firms that utilize strategic and tactical actions will better discern the type of market change and its potential effects. There is a possibility that businesses with more insight from social media might perform better than their counterparts. Here, we proposed the following hypothesis:

*H1*: Knowledge acquisition from social media has a significant impact on brand innovation strategy on social media.

### Using Social Media for Market Orientation and Brand Innovation

A market-oriented organization discovers and understands the needs of its customers. In other words, the development of new technologies is driven by latent market needs, both internal and external, including the requirements of lead customers or users. For many scholars (i.e., Hanusch and Tandoc, 2019), it is difficult to obtain accurate information about latent customer needs. Customers may not know their preferences for innovative products in potential markets.

It is believed that the development of new products, services, and ideas will originate from addressing consumers’ latent needs. Mpandare and Li (2020) stated that proactive market orientation emphasizes understanding customers’ needs as a process that starts from the outside. An innovative social media strategy can be launched by leveraging proactive market orientation and customer knowledge.

Social media brand innovation requires a proactive market orientation. In their study of market orientation and innovation, Levine and Zahradnik (2012) pointed out that market orientation promotes radical innovation offline. Social media channels appear to have the same effect in today’s context. Focusing on long-term developments is an essential element of proactive market orientation since it is related to market information and thus can lead to radical product innovations. Actions requiring continuous awareness of latent customer needs can then be achieved by discovering, understanding, and innovatively satisfying them (Mitchell et al., 2010; Awan et al., 2021b).

An approach is known as “responsive market orientation” aims to identify and meet customers’ expressed needs (Ferrucci, 2020). The interaction between users on social media and their use of online reviews and blogs demonstrate that users are adept at expressing their opinions and using products and services. According to research, an orientation toward responsive markets can lead to incremental rather than drastic improvements in products or services. Tajurahim et al. (2020) discussed that customer centricity is positively related to innovation in some studies. It does not seem that market orientation negatively impacts China’s level of innovation. The explanation for this can be found in the study of Khamaludin et al. (2022), who explains that customers’ expressed needs can be met both explicitly and implicitly. Chinese emerging market consumers have many expressed needs that are not met.

Gul et al. (2021) described market orientation as an organization’s ability to combine or integrate its skills and resources in a way that adapts quickly. Poole has created a correlation between the development of a new product, the direction of the market, and the company’s export capacity (Kovacova et al., 2020). Market trends such as the expansion of market intelligence businesses, the transmission of information to other departments, and a company’s overall response are all taken into account when forecasting the market’s future direction. As a result of Lu et al. (2020) study, people have developed a greater interest in the market’s direction. Competitive advantage has been thoroughly examined, and a more comprehensive technique for quantifying it has been developed. Inter-functional coordination is critical, as are competition and customer orientations. These are only a few of the aspects that contribute to a market-oriented strategy. Kovacova and Lewis (2021) refer to this as market orientation when discussing or describing anything intangible. Being aware of your competitors, your consumers, and their activities can provide you a competitive edge. This resource is inextricably linked to the rest of the globe.

Cai et al. (2015) emphasized that Chinese typesetting characters by hand before laser technology was developed were a bothersome task. A series of lasers was used to typeset Chinese characters, a technological breakthrough. We can create more radically innovative solutions if we understand the customer’s needs despite no existing solutions if we understand the customer’s needs. Hence, we proposed the following hypotheses:

*H2a*: Proactive social media market orientation has a significant impact on brand innovation strategy on social media.

*H2b*: Responsive social media market orientation has a significant impact on brand innovation strategy on social media.

### Strategic Capability and Brand Innovation on Social Media

In today’s market, staying abreast of the changing landscape of online technology is essential. A company needs to react rapidly to market changes, technological uncertainties, and competitors’ action\s if it is successful (Habibi et al., 2015; Awan et al., 2021c). The process of building firm-specific advantages, which enhance the firm’s strategic benefits, uses both tangible and intangible resources (knowledge and assets). The firm’s strategic direction encompasses exploring new opportunities or utilizing existing products and expanding into other areas in which it is active. Resources determine how strategic capabilities are implemented. According to Herrero et al. (2018), an organization’s strategic capabilities are limited by its resources. Levine and Zahradnik (2012) described social media strategic capability as a unique resource, which is similar to a resource that represents a unique competitive advantage, as well as helping to facilitate strategic value creation since it provides the ability to manage resources, a characteristic of capabilities of this kind. By acquiring and integrating resources, firms can enhance their innovation capabilities (Mohsin et al., 2021a).

Companies with more substantial strategic capabilities in social media have better access to information and technology critical to success. Such firms will benefit from such capabilities by gaining access to unique data, technology, and support and responding to environmental changes more proactively (Saavedra et al., 2014; Jamil et al., 2021a). It can take a while for start-ups without affiliations and limited resources to build such a capability. While trial-and-error can be expensive, the knowledge it provides can assist an organization in identifying and assessing useful information for innovation in a proactive manner once it is complete (Odoom and Mensah, 2019; Li et al., 2021). A turbulent environment can enable new, innovative activities by reallocating resources based on such information. In discussing the sources of help and social capital derived from networks and, particularly, social media knowledge, we conclude that organizations can better access and integrate resources using social media networks and be more innovative (Arrigo, 2018). Hence, the following hypothesis was proposed as:

*H3*: Strategic capability on social media has a significant impact on brand innovation strategy on social media.

### Moderating Role of Strategic Capability

Muninger et al. (2019) proposed that an organization’s sustainable competitive advantage may originate from its resources and its ability to integrate and transform them. In addition, these researchers state that non-tangible external resources can contribute to internal capital only if they are transferrable. In addition to organizing and coordinating different resources and functional units, Tarsakoo and Charoensukmongkol (2020) observed that strategic capability can only benefit an organization’s innovation agenda without adequate resources. Strategic capability is essential to ensuring a firm’s competitiveness; it plays a significant role in making strategic decisions, especially innovation. Firm-specific capabilities can be supported and promoted *via* better strategic social media capabilities (Garrido-Moreno et al., 2020; Mohsin et al., 2021b). By acquiring social media knowledge, companies can obtain valuable information and other resources to develop innovative solutions and use this information to achieve their strategic goals. Companies use social media to interact and conduct business among themselves and improve productivity and efficiency. Social media strategists need a higher level of strategic capability if they are going to increase brand innovation through social media. Zhang and Zhu (2021) argued that a strategic decision can be made within an organization efficiently and precisely under social media strategic capabilities, based on the organization’s resources and ability to convert knowledge into a competitive edge.

A strategic approach to resource allocation and product design also increases the likelihood of successful brand innovation. Adoption is accomplished by absorbing and applying new external resources, which stimulates the development of new product variants and the exploration of new capabilities. Our study indicates that companies’ ability to integrate and use external resources (such as technology resources) in combination with a broad range of social media strategic capability with vast information will likely increase their ability to discover and experiment with novel brand innovation opportunities through social media (Jamil et al., 2021b; Ngammoh et al., 2021).

Researchers examine the relationship between market demand and innovation, looking at internal technological capabilities and the uncertainty of market needs (Wang et al., 2017). They contend that both of these factors contribute to innovation. Radical innovations requiring significant investment resources require both technology and investment capabilities. When a firm competes, these commitments determine its survival and development. It is also vital to have strategic capabilities. Trying to anticipate latent customer needs in a proactive market orientation by focusing on unfamiliar information and knowledge (Mention et al., 2019). To achieve more significant results, proactiveness in the marketplace and brand innovation can be brought together with effective social media strategic capabilities owing to better alignment and focus (Sarfraz et al., 2021; Zhang and Zhu, 2021). We expect that China’s social media market will be a dynamic and turbulent one that will require superior social media capabilities to drive brand innovation and enhance proactive market positions effectively. Consequently, proactive market orientation will significantly impact brand innovation where social media strategies are employed (Garrido-Moreno et al., 2020).

We further propose that companies with immense social media strategic capability better understand their available resources and how they should be allocated and integrated, which will cause improved brand innovation through a market-responsive orientation (Foltean et al., 2019; Odoom and Mensah, 2019). Although social media strategic capabilities may improve proactive and reactive actions, they can also directly impact proactive/reactive market orientation and brand innovation. It may moderate market orientation and innovation to a greater extent because social media has a short-term focus, therefore aligning well with social media strategic capability (Maghsoudi Ganjeh et al., 2019; Naseem et al., 2021). Social media strategic capabilities are also emphasized in the rapidly changing market context. Social media strategies can still assist these companies in achieving proactive market orientation, however, as they give them an increased chance of identifying latent consumer demands. A proactive marketing strategy involves selecting high-return projects (Liu et al., 2021). The best way to do this is to identify latent needs that opportunistic companies can exploit in social media. Through social media development, the integration of expressed knowledge, and a solid market-oriented approach, brand innovation efforts can also be enhanced. With the help of social media-related strategic capabilities, firms can leverage existing customer knowledge, information, resources, and knowledge to improve their performance by focusing resources quickly and allocating resources to the right project (Tarsakoo and Charoensukmongkol, 2020). Hence, we proposed the following hypothesis:

*H4a*: Strategic capability on social media moderates the relationship between knowledge acquisition from social media and brand innovation on social media.

*H4b*: Strategic capability on social media moderates the relationship between proactive social media market orientation and brand innovation on social media.

*H4c*: Strategic capability on social media moderates the relationship between responsive social media market orientation and brand innovation on social media (see Figure 1 for all relationships).

**Figure 1:** Conceptual framework.

### Conceptual Framework

#### Research Methodology

This study designed a questionnaire according to the hypotheses stated above. The participants in this study were online technology firms in China. Based on the technology commercialization practices of firms and social networks, we included our primary sampling frame to invite LinkedIn China, Weibo China, WeChat China, RenRen, Ozone and company websites. We approached each firm’s principal founder or senior managers to collect accurate data utilizing an online questionnaire-survey approach. Online questionnaires have the following advantages (Tan and Teo, 2000): (1) sampling is not restricted to a single geological location, (2) lower cost, and (3) faster questionnaire responses. Before the final analysis, a pilot study with 100 participants was carried out. Since providing recommendations, revisions were made to the final questionnaire to make it more understandable for the study’s respondents. To ensure the content validity of the measures, three academic marketing experts analyzed and made improvements in the items of constructs. The experts searched for spelling errors and grammatical errors and ensured that the items were correct. The experts have proposed minor revisions to market orientation and brand innovation strategy items and advised that the original items be maintained. A total of 853 questionnaires were returned from respondents. There were 853 appropriate replies considered for the final analysis.

#### Measures

The study used items established from prior research to confirm the reliability and validity of the measures. All items are evaluated through five-point Likert-type scales where “1” (strongly disagree), “3” (neutral), and “5” (strongly agree).

##### Dependent Variable

To get a response about brand innovation strategy, we used four items adapted from the prior study of Cheng and Shiu (2008), and the sample item is “Brand innovation using social media is a breakthrough innovation practice.”

##### Independent Variables

To get the response about knowledge acquisition, we used five items adopted from the prior study of Zhou and Li (2012), and the sample item is “Our company has a process for continuously collecting information from customers using social media.” Furthermore, to get a response about proactive orientation, we used four items adapted from the previous study of Narver et al. (2004). The sample item is “We help customers anticipate developments in the markets using social media.” Moreover, to get a response about responsive orientation, we used three items adopted from the prior study of Narver et al. (2004). The sample item is “We measure customer satisfaction systematically and frequently using social media.”

##### Moderating Variables

We used strategic capability as moderating variables in this study. To get a response about strategic capability, we used four items adapted from the prior research of Croteau and Raymond (2004), and the sample item is “My organization owns future competitive flexibility in social media.”

## Results

### Measurement Model (Outer Model)

The measurement’s model analysis explains how dimensions of latent variables are dignified regarding their measurement properties and perceived (observed) items. This specific section highlights the evaluation of the outer model (measurement) by assessing the internal consistency, item’s reliability, discriminant validity, and convergent reliability (Henseler et al., 2009; Hair et al., 2011; Usman Shehzad et al., 2022).

Inclusively 20 items to explain the four constructs of the model. Using the PLS algorithm for all reflective constructs was accomplished. The SMART-PLS algorithm assessed the reflective scale’s reliability through convergent reliability and discriminant validity estimations. The following model depicts latent variables (circles), and their measuring items (rectangles) appear in Figure 2.

**Figure 2:** Measurement model.

These results show that all latent variables in the model are reflective by nature. Results define it that all-inclusive quality of the reflective variable’s measure of PLS loadings, Cronbach’s alpha, constructs AVE and composite reliability, shown in Table 1. By evaluating the first-order construct, the item’s loading was assessed (Table 1). Regarding Knowledge Acquisition from Social Media, it consisted of five items. The outer loadings fluctuated from 0.651 to 0.737 for concerned items, and all items are significant at the level of 0.5, shown by the *t-*value results. Proactive Social Media Market Orientation with no dimension, but it comprises four items. The outer loadings fluctuated from 0.882 to 0.746 for concerned items, and all items are significant, as shown by the *t-*value results. Three items with no dimension assessed responsive Social Media Market Orientation. The outer loadings fluctuated from 0.711 to 0.711 for concerned items, and all items are significant at the level of 0.5, shown by the *t-*value results. Four items assessed social Media Strategic Capability. It has no dimension as well. The outer loadings fluctuated from 0.790 to 0.878 for concerned items, and all items are significant at the level of 0.5, shown by the *t-*value results. Four items assessed social Media Brand Innovation. It has no dimension as well. The outer loadings fluctuated from 0.785 to 0.858 for concerned items, and all items are significant at the level of 0.5, shown by the *t-*value results.

**Table 1:** Measurement statistics of constructs.

Constructs, Dimensions, Items	Item loading	AVE	CR	Α
Knowledge Acquisition				
KAS2	0.878	0.904	0.924	0.636
KAS3	0.759			
KAS4	0.874			
Proactive Market Orientation				
PSMO2	0.801	0.816	0.854	0.595
PSMO3	0.648			
PSMO4	0.848			
Responsive Market Orientation				
RSMO1	0.868	0.831	0.887	0.663
RSMO2	0.810			
RSMO3	0.581			
Strategic Capability				
SMBI1	0.813	0.882	0.919	0.740
SMBI2	0.821			
SMBI3	0.798			
SMBI4	0.813			
Brand Innovation				
SMSC1	0.878	0.840	0.889	0.689
SMSC2	0.774			
SMSC3	0.868			

### Convergent Validity

Additionally, the discriminant validity of the framework was tested using Fornell and Larcker criterion (Sarstedt et al., 2014). The Fornell Lacker criteria suggest that the square root of the AVE values for all constructs should be greater than the correlation among the pair of constructs (Fornell and Larcker, 1981). The model is discriminately valid when the criteria are fulfilled, as shown in Table 2.

**Table 2:** Discriminant validity.

	KAS	PSMO_	RSMO	SMBI_	SMSC
KAS	0.880				
PSMO_	0.867	0.870			
RSMO	0.658	0.646	0.763		
SMBI_	0.762	0.726	0.671	0.868	
SMSC	0.860	0.753	0.652	0.840	0.841

*The square root of AVE’ is visible on the main diagonal; correlations are lower left*.

### R-Square

The hypothesis was tested using 5000 bootstraps. R-square and Q-square, as suggested by, were used to assess the structural model (Hair et al., 2016). To be termed moderate, the coefficient of determination (R-square) must have a value over 0.33 (Chin, 1998). For Social Media Brand Innovation, the R-square is 73.8 per cent. The panel also backed up the Q-positive square’s results. The predictive significance of the model was evaluated using the “cross-validated redundancy” Q2 test (Hair et al., 2014). Q2’s value must be bigger than “zero” to be considered acceptable. Greater than 0 is seen in the Q squared values. Q2 values of exogenous construct demonstrate the accuracy of the study framework in predicting outcomes (Hair et al., 2016). According to the researchers, the prediction accuracy of a model may be evaluated using R2 (Henseler et al., 2015; see Table 3).

**Table 3:** Predictive relevance of the model.

	R-Square	R-Square Adjusted
Brand Innovation	0.738	0.741

### Hypothesis Testing

This study evaluates the significance of relationships by using Bootstrapping at 5000 with a replacement sample (Hair et al., 2016). The results indicate that knowledge acquisition from social media significantly impacts brand innovation strategy ( *β* = 0.643, *t* = 12.284, *p* = 0.000); these findings support the H1. The proactive social media market orientation significantly affects brand innovation strategy on social media ( *β* = 0.047, *t* = 3.162, *p* = 0.002); results approve the H2a hypothesis. Responsive social media market orientation significantly impacts brand innovation strategy on social media, where the results are significant with ( *β* =0.119, *t* = 4.542, *p* = 0.000), which support H2b. On the other side, strategic capability on social media has a significant impact on brand innovation strategy on social media with significant ( *β* =0.129, *t* = 0.128, *p* = 2.224), these findings support the H3 (see Table 4 and Figures 3, 4).

**Table 4:** Result of structural model and hypotheses testing.

	Original Sample (O)	Sample Mean (M)	Standard Deviation (STDEV)	T Statistics (|O/STDEV|)	Values of *p*
KAS - > SMBI_	0.643	0.641	0.052	12.384	0.000
PSMO_ - > SMBI_	0.047	0.045	0.015	3.162	0.002
RSMO - > SMBI_	0.119	0.119	0.026	4.542	0.000
SMSC - > SMBI_	0.129	0.128	0.058	2.224	0.026

**Figure 3:** PLS bootstrapping with values of *p*.

**Figure 4:** PLS bootstrapping with values of *t*.

### Testing the Moderating Effect

A moderating impact happens when a third factor (so-called mediator) decreases or improves the quality or direction of the relationship between independent and dependent variables (Lindley and Walker, 1993). A moderator variable communicates under what conditions independent variable impacts on dependent variable (Baron and Kenny, 1986). Considering a causal variable, a moderator is similar to an independent variable. A few measurable procedures have been predicted in testing moderating impacts, contingent upon whether the moderator is categorical or continuous.

When the exogenous variable effect on endogenous variable depends upon the estimations of another variable, which moderates the link, Vinzi et al. (2010) evaluate different approaches for testing moderation in Smart-PLS-SEM far as their relevance to statistical power and reflective and formative measure. Institutional pressure moderates the relationship between HR practices and proximal factors.

The association between knowledge acquisition from social media, proactive social media market orientation, responsive social media market orientation, strategic capability on social media, and social media and brand innovation on social media are shown in the table. All the moderating effects are positive and significant. It offers significant results consistent with the previous research; the results show that strategic capability on social media influences the relationship between knowledge acquisition from social media, proactive social media market orientation, responsive social media market orientation, and brand innovation on social media are significantly and positively (see Table 5).

**Table 5:** Hypothesis testing result moderating effects.

	Original Sample (O)	Sample Mean (M)	Standard Deviation (STDEV)	T Statistics (|O/STDEV|)	Values of *p*
KAS^*^SMSC_ - > SMBI_	0.073	0.072	0.014	5.293	0.000
RSMO^*^SMSC_ - > SMBI_	0.121	0.122	0.023	5.248	0.000
PSMO^*^SMSC - > SMBI_	0.064	0.064	0.020	3.206	0.001

#### Moderating Effect 1

According to Figure 5, strategic capability on social media moderates the relationship between knowledge acquisition from social media and brand innovation on social media. Thus, Hypothesis H4a is supported.

**Figure 5:** Interaction effect of strategic capability on social media and knowledge acquisition from social media predicting brand innovation on social media.

#### Moderating Effect 2

In Figure 6, strategic capability on social media moderates the relationship between proactive social media market orientation and brand innovation. Thus, Hypothesis H4b is supported.

**Figure 6:** Interaction effect of strategic capability on social media and proactive social media market orientation predicts brand innovation on social media.

#### Moderating Effect 3

According to Figure 7, strategic capability on social media moderates the relationship between responsive social media market orientation and brand innovation on social media. Thus, Hypothesis H4c is supported.

**Figure 7:** Interaction effect of strategic capability on social media and responsive social media market orientation predicts brand innovation on social media.

## Discussion

This paper explores market orientation, social media knowledge, brand innovation, and social media strategic capability and empirically tests them in China’s dynamic social media environment. We propose that social media learning, including market orientation and knowledge acquisition, fosters brand innovation complemented by social media strategic capabilities. In the following section, we discuss the study’s significant findings in detail and discuss the contribution and implications.

According to the results, the factors associated with learning-centered brand innovation can be divided into several groups. The path coefficients indicate that the most influential construct on brand innovation is social media knowledge acquisition. The influence of responsive market orientation, and proactive market orientation, is also significant this result is parallel with the previous study of Odoom and Mensah (2019). For researchers, market orientation and knowledge acquisition boost the focus firm’s competitiveness because they enable it to co-create value with internal and external stakeholders. In light of this nuanced finding, companies should use social media as their primary source of knowledge acquisition. It stands to reason that the new online technology company will have to allocate its limited resources more efficiently due to this finding.

The degree of radical brand innovation on social networks is positively associated with proactive and responsive market orientations. These studies provide evidence that proactive market orientation and innovation are related, in line with earlier studies conducted in a traditional offline context (Cai et al., 2015). Innovative product and service creation are facilitated by this model, which can enable social media ventures to remain competitive. A market orientation strategy can, contrary to conventional wisdom, contribute to brand innovation, as evidenced by the results of this study. Social media allows for more comprehensive searches and identification of customers’ needs, expressed and latent (or unexpressed). The new rules of the competition and strategic behavior presented by social media should be considered by online technology companies.

Chinese online technology firms benefit from a market-driven focus when developing an innovation strategy that leads to radical change. It has been found that the results of this study conflict with most theories developed in Western contexts; however, transitional economies are more volatile and dynamic, which is exacerbated by the presence of social media in this case. Study results confirm this viewpoint by demonstrating that firms in China can sustain rapid and stable growth by focusing short-term on expressed needs during the country’s transitional economic phase. It is critical to focus on customer needs that cannot be described to advance radical innovation to a new level (Migdadi, 2021). Our study found that both the transitional country effect and the social media context are influential in brand innovation strategies in distinct ways.

### Theoretical Implications

Three new contributions are made to the literature by studying social media branding. On the one hand, we show how proactive and responsive marketing orientation can be applied to social media. Our work offers new perspectives on market orientation and brand innovation strategy by extending the literature and testing key assumptions. In general, radical innovations are more likely to emerge in companies with a proactive orientation to the market. Several conclusions can be drawn from our study, including that marketing orientation types and brand innovation are interconnected, as well as the possibility that strong social media strategic capability can lead to a more radical approach to brand innovation. Resource constraints often determine the use of one orientation over the other (Tarsakoo and Charoensukmongkol, 2020). This study demonstrates that organizational ambidexterity may be moderated by social media strategic capability.

In addition, this study adds empirical support to the theory of social capital by demonstrating that the capability of social media to assume a strategic role in knowledge acquisition is an important mediating factor. Social media can improve the process of knowledge acquisition by reducing the negative effects of poor organizational infrastructure, especially given the high-risk and resource-consuming nature of innovation (Hafez, 2021). These reciprocal relationships produce new opportunities and ideas based on information and knowledge shared by these businesses. A firm’s brand innovation strategies can also be made less risky and resource-constrained by these strategies. Various types of information and resources are transformed by social media strategic capabilities to enhance the competitive advantage of online technology firms. Thus, firms have become more capable of managing dynamic resources, enabling them to leverage the skills and knowledge they have gained from social networks to augment their social capital, ultimately leading to better brand innovation performance.

### Managerial Implications

The study finds that new online technology ventures will positively influence brand innovation through social media strategic capability. We believe that using social media knowledge in social media marketing and innovation management is a sensible approach for making changes and transforming an organization. Firms with a social media strategy capability may be better able to identify opportunities and adjust accordingly during the brand innovation process (Wang et al., 2017). The only way to achieve this is to use a market-focused approach and acquire continuous knowledge from social media. The company could achieve its goals through many methods, such as using a more viable brand innovation process, implementing new technology, or aiming for a new market after the changes are implemented. Businesses can disrupt markets and eliminate existing practices more effectively with social media. Marketers can stay on top of social media by following the framework and guidelines presented in our study.

### Limitations and Future Research Directions

This study has a few limitations. First of all, an online setting was used to test our theoretical framework. Therefore, our results cannot be generalized to other settings. Time and financial concerns also limited our study, so we collected data from one location. A more in-depth understanding of our approach could also be gained by applying our results to other economies. Research in the future should examine these variables and different innovation types, including incremental innovation.

## Data Availability Statement

The raw data supporting the conclusions of this article will be made available by the authors, without undue reservation.

## Author Contributions

All authors listed have made a substantial, direct, and intellectual contribution to the work, and approved it for publication.

## Funding

This research was supported by a key project of Anhui Social Sciences Innovation and Development research project (grant no. 2021CX064).

## Conflict of Interest

The authors declare that the research was conducted without any commercial or financial relationships that could be construed as a potential conflict of interest.

## Publisher’s Note

All claims expressed in this article are solely those of the authors and do not necessarily represent those of their affiliated organizations, or those of the publisher, the editors and the reviewers. Any product that may be evaluated in this article, or claim that may be made by its manufacturer, is not guaranteed or endorsed by the publisher.
